The article "pH Dependent Molecular Self-Assembly of Octaphosphonate Porphyrin of Nanoscale Dimensions: Nanosphere and Nanorod Aggregates" was retracted in 2021. Reasons: manipulated images; unreliable results or conclusions; no approval from an author.

# pH Dependent Molecular Self-Assembly of Octaphosphonate Porphyrin of Nanoscale Dimensions: Nanosphere and Nanorod Aggregates

**DOI:** 10.3390/ijms12031464

**Published:** 2011-02-24

**Authors:** Sheshanath V. Bhosale, Mohan B. Kalyankar, Santosh V. Nalage, Cecilia H. Lalander, Sidhanath V. Bhosale, Steven J. Langford, Ruth F. Oliver

**Affiliations:** 1 School of Chemistry, Monash University, Wellington road, Clayton Victoria 3800, Australia; E-Mails: kalyankar.mb@rediffmail.com (M.B.K.); cecilia.lalander@monash.edu (C.H.L.); steven.langford@monash.edu (S.J.L.); ruth.oliver@monash.edu (R.F.O.); 2 Department of Organic Chemistry, North Maharashtra University, Jalgaon 425 001, India; E-Mail: snalage@yahoo.com (S.V.N.)

**Keywords:** molecular self-assembly, porphyrin, aggregation, AFM, TEM

## Abstract

Self-assembled nanostructures of zwitterionic octaphosphanatoporphyrin **1**, of either nanoparticles or nanorods, depending on small changes in the pH, is demonstrated based on the J-aggregates. Porphyrin **1** self-assembled into nanosphere aggregates with a diameter of about 70–80 nm in the pH range 5–7, and nanorod aggregates were observed at pH 8.5. Hydrogen bonding, *π*-*π* stacking and hydrophilic interactions play important roles in the formation of this nanostructure morphology. Nanostructures were characterized by UV/Vis absorbance, fluorescence, atomic force microscopy (AFM) and transmission electron microscopy (TEM). This interesting pH dependent self-assembly phenomenon could provide a basis for development of novel biomaterials.

## 1. Introduction

Porphyrins, particularly natural *i.e.*, chlorophylls and the protoporphyrin IX, contain hydrophobic, rigid, apolar and polar parts [1]. This characteristic prevents crystallization and favors self-aggregation [2]. Such supramolecular self-assemblies are of interest for polymeric porphyrin wires for long range energy and electron transport [3]. In contrast, symmetric tetraphenylporphyrins (TPPs) lack this diversity of functional groups and have a high tendency to crystallize. However, water-soluble symmetric TPP derivatives [4,5] form nanostructures or form well-defined Langmuir-Blodgett monolayers on smooth solid surfaces [6], and TPP derivatives carrying long side chains with water-soluble groups produces fibrile structures at low pH [7,8]. Nevertheless, recently we have shown that substituted protoporphyrin (IX) with triethylene glycol [9], which shows good solubility in organic solvents, produces well defined tunable nanostructures from varying solvent mixes.

Phosphonatoporphyrin were first developed as building blocks for porphyrin towers on silicon or gold electrodes for electrochemical investigations, in such a case zirconium-(IV) was first applied as a cement between phosphonate groups and led to broad rocks, instead of ill-defined monomolecular aggregation [10]. Self-assembly of phosphonatoporphyrin with more flexible chains was proven to result in formation of ill-defined monomolecular aggregates [11]. There are only few reports of porphyrin vesicles from charged and/or amphiphilic porphyrins [12–19]. Nanoscaled three-dimensional aggregates of supramolecular porphyrin arrays have been explored and their non-specific intermolecular interactions have been described. A porphyrin derivative substituted by four cartenoid molecules (“bixin”) spontaneously formed vesicles in water, as observed by Fuhrhop and co-workers [18]. Vesicles of meso-tetrakis-[(bixinylamino)-*o*-phenyl] porphyrin formed in water at pH = 9 can remain essentially intact even on dry solid surfaces [18,19]. Systematic studies on the anionic substituent are desired to further develop the research scope of the zwitterionic self-assembly of porphyrins. For the J-aggregate formation, the electrostatic interactions between the positively charged porphyrin core and the negatively charged groups play an important role. However, studies along these lines are still limited [4,5]. Nevertheless, in our earlier work, we have demonstrated synthesis of novel octaphosphanatoporphyrin (OctaPhosPor) **1** [20], and its cofacial reversible self-assembly with cyclam, which yields micrometer long monomolecular nanowires. We speculated that self-assembly was modulated by intermolecular hydrogen bonding of the amino groups of cyclam with phosphonato moieties of **1**. In this present study, we report pH dependent self-assembly of zwitterionic OctaPhosPor **1** in water, and the displacement of peripheral phosphanato (anionic) groups of porphyrins is shown to have a major effect on the aggregation behavior.

## 2. Results and Discussion

Porphyrin **1** is equipped with two phosphonate moieties on the *meta*-positions of each phenyl group with methylene bridges (Figure 1). Short flexible spacers, *i.e*., methyl, were found to be necessary to achieve good solubility of the phosphonate esters in organic solvents and phosphonate salts in water. By manipulating pH, we show that supramolecular adducts form in solution and further stabilize by H-bonding to form nanospheres and nanorods in water (Figure 1). To the best of our knowledge, phosphonate moieties on porphyrin forming nanoscale aggregates have not yet been reported.

We hypothesize that pH dependent assemblies of OctaPhosPor **1** were obtained via three protonation steps (see Figure 1b): (1) first protonation of the phosphonate groups (p*K*a = 8.0), (2) protonation of the core nitrogen atoms (p*K*a = 5.6), and (3) second protonation of the phosphonate groups (p*K*a = 3.0). It is expected that the second protonation step, leading to a zwitterionic form, might induce aggregation. On the other hand, the first protonation step produces a nonzwitterionic species that is able to aggregate. In the latter case, in addition to *π*-*π interactions*, hydrogen bonds involving the phosphonic groups might also foster self-assembly. In this case, dimers of porphyrins interact axially through *π*-*π* stacking and laterally by means of strong edge-to-edge hydrophobic contacts. The whole structure may further stabilize by hydrogen bonding of phosphonato groups. Our experimental results agree with previous literature assignments [11]: OctaPhosPor **1** is (i) a monomer at pH > 9.0, (ii) a spherical particle aggregate at pH range 5–7, and (iii) higher aggregates are observed in the pH range 7–9. The stability of the particles and tubular aggregates made of porphyrins is presumably caused by an ordering of the porphyrins by *π*-*π* interactions and by hydrogen bridges between partly protonated phosphonate groups in water at higher pH. The aggregation behavior of **1** in aqueous solution, as a function of pH, has been studied by means of UV/Vis, fluorescence emission spectroscopy, atomic force microscopy (AFM) and transmission electron microscopy (TEM) techniques.

### 2.1. UV/Vis Absorption and Fluorescence Spectroscopy

Typically OctaPhosPor **1** is readily soluble in water at pH 9.0 and the corresponding UV/Vis spectrum exhibits an intense Soret band at 418 nm (ɛ = 2.56 × 10^5^ L M^−1^ cm^−1^), together with four weaker Q-bands at 516, 558, 584, and 639 nm (Figure 2, broken curve). In fact, at pH 5.5, the most prominent band in the absorption spectrum is red-shifted with respect to that of the species existing at basic pH 9.0. At pH 5, absorption of **1** shows a red-shifted Soret band at 440 nm with vanishing of three Q-bands and appearance of a red-shifted Q-band at 656 nm (Figure 2, solid curve). The appearances of such characteristic absorption bands indicate the formation of J-aggregates. The “lack” of the Soret band of the protonated form (418 nm, monomer porphyrin band) can be attributed to the aggregation phenomena [12–18]. The effect of changing pH has been investigated in the pH range 3–11 (Table 1). The absence of the Soret band of the protonated form strongly suggests that the higher aggregate presiding over the hierarchy is that formed at a pH close to 6–8.

Furthermore, fluorescence emission of OctaPhosPor **1** shows two bands at 651 and 718 nm at pH 8.5 upon excitation at λ_max_ = 418 nm. In sharp contrast, the fluorescence decreases with a decrease in pH with a slight bathochromic shift, which also indicates aggregation behavior of **1** (Figure 3). At pH 9–11, porphyrin appear to be in monomeric form, and in acidic pH (in the range 5–9) fluorescence quenching was observed. Such fluorescence quenching may be due to the self-aggregation of porphyrins at such pHs [12–18].

To support this hypothesis, we have characterized self-assembly of **1** at different pHs from 5–9, by employing atomic force microscopy (AFM) and transmission electron microscopy (TEM) techniques.

### 2.2. Atomic Force Microscopy and Transmission Electron Microscopy

Porphyrin **1** (10^−4^ M) gives nanospheres with a mean diameter of *ca.* 70–80 nm and a height of *ca.* 30 nm at pH 7.0 in water (Figure 4). The mean diameter of the particles (75 nm) is significantly larger than the molecular dimension of **1** (*ca.* 2.2 nm), hence nanoaggregates should be vesicular aggregates rather than micellar aggregates. Furthermore, transmission electron microscopy (TEM) gave clear evidence of formation of vesicular aggregates of porphyrin **1**. TEM shows well-defined completely regular and isolated pattern of aggregated nanospheres of **1** with a mean diameter of 70–100 nm (Figure 4d). The TEM images are in excellent agreement with the results obtained from AFM, with respect to the size and diameter of these nanospheres measured. In addition, it can be seen from the TEM images that the spherical particles are completely dispersed and do not tend to associate with each other.

At pH 8.5, **1** produces not only the common particular aggregates but also regular parallel-lying self-organized nanorods (Figure 5). The AFM images showed that most of the tubules were surrounded by disordered and mobile patches of flat-lying porphyrins (Figure 5a). Occasionally these tubules showed some crystalline order at one end and the other end narrow. TEM examination of the same sample prepared from a dilute solution of **1** at pH 8.5 revealed the presence of well-defined rod like nanoaggregates with a diameter of ∼15 ± 3 nm and of several nanometers in length (600–900 nm) as shown in Figure 5b. Interestingly, the change to pH < 8.0 reduces the average size of the aggregates and leads to the formation of assemblies with short nanorods.

That self-assembly only occurs in pH 5–9 was confirmed by fluorescence spectroscopy, as in the pH range 3–5, the emission of **1** was diminished, which may be due to the protonation of phosphonate end groups and the two nitrogen atoms of the core. AFM clearly shows formation of larger aggregates *i.e*., nanosheets at pH values above 10 and below pH 5 as shown in Figure S1 and S3, respectively.

## 3. Experimental Section

### 3.1. Octaphosphanato Porphyrin **1** Synthesis

Synthesis and characterization of OctaPhosPor **1** was described previously [1].

### 3.2. Standard Solution of Octaphosphanato Porphyrin **1**

Stock solutions (concentration 1 × 10^−3^ M) of **1** were made in water at pH 7.0. For spectral measurements, this solution was injected each time with 2 mL of water (varying pH) in a cuvette using a micropipette.

### 3.3. UV-Vis Absorption Spectroscopy

Stock solutions (concentration 1 × 10^−3^ M) of **1** were made in water (pH 7.0). A 0.2 mL aliquot of the stock solution was transferred to several different volumetric flasks in water at varying pH 3–11, each of 2 mL volume. The solutions were allowed to equilibrate for 2 h prior to the spectroscopic measurements. The most prominent features are a reduction in the peak intensity along with a significant red shift of the absorption maximum and a loss of the fine structure.

### 3.4. Atomic Force Microscopy (AFM) of **1**

The samples were characterized using an Atomic Force Microscope (AFM) from Agilent Technologies (5500 AFM). Micromach Ultrasharp probes with silica wafer coating for enhanced reflectivity (NSC15/AIBS), with a typical resonance frequency of 325 kHz and a force constant of 40 N/m, were used for imaging. Sample of OctaPhosPor **1** were prepared by spin-coating the freshly prepared solution (1 × 10^−4^ M in water, at varying pH 3 to 11) onto silica coating at 2000 rpm. The particle diameter and height determination was performed by measuring the mean horizontal distance and height of particles.

### 3.5. Transmission Electron Microscopy (TEM) of OctaPhosPor **1**

TEM measurements were performed on an electron microscopy Igor 1200EX, operating at an accelerating voltage of 80 kV. 0.5 μL freshly prepared sample solution (1 × 10^−4^ M in water at different pH values) was dropped onto a TEM grid (400-mesh copper grid coated with carbon) and the solvent was allowed to evaporate before introduction into the vacuum system. Negative staining was performed by addition of a drop of uranyl acetate onto the carbon grid. After few minutes, remaining solvent was removed by tapping with filter paper and images were collected.

## 4. Conclusions

In this paper, we have shown that by tuning the pH systems through the formation of complementary hydrogen bonds it is possible to promote the formation of nanospheres and nanorods of phosphonato porphyrin in water. The formed self-assembled nanostructures, *i.e*., nanospheres and nanorods, were stable enough to be investigated in solution via UV/vis, fluorescence spectroscopy and visualized through AFM and TEM microscopy. We are also currently producing porphyrin phosphonate nanoscale aggregates from zinc and tin(IV) complexes in order to measure electric conductivities of cation and anion π-radical stacks [21].

## Figures and Tables

**Figure 1.** **(a)** Schematic representation of the self-assembly of the OctaPhosPor **1** into: nanosphere aggregates at pH 5–7, and further aggregation of **1** into nanorods at pH 7–9 in water; **(b)** protonation and aggregation mode of OctaPhosPor **1**.

**Figure 2.** Absorption spectrum of OctaPhosPor **1** (1 × 10^−4^ M) at pH 9.0 (broken curve) and 5.0 (solid curve), inset figure shows as an expansion of Q-bands (490–690 nm).

**Figure 3.** OctaPhosPor **1** shows a pH dependent (10.4–3.0) change in fluorescence spectrum at a concentration of 1 × 10^−4^ M, λ_ex_ at 418 nm.

**Figure 4.** Atomic force microscopy (AFM) height images of OctaPhosPor **1** (10^−4^ M) upon spin-cast on silicon wafer plate after the solvent has evaporated, gives nanospheres in water at pH 7.0: (**a**) height image (scale bar = 1 μm); (**b**) magnified view of height image a (scale bar = 400 nm); (**c**) height image (scale bar = 1 μm); (**d**) Transmission electron microscopy (TEM) micrograph of **1** on holey, carbon-coated copper grids (scale bar = 100 nm); (**e**) high magnification of d; and (**f**) cross-section analysis magnified region from image c, provides a mean diameter of *ca.* 75 nm and a height of 30 nm.

**Figure 5.** (**a**) Atomic force microscopy (AFM) height images of **1** (10^−4^ M) upon spin-cast on silicon wafer plate after the solvent has evaporated; Inset = high magnification of AFM image (**b**) Transmission electron microscopy (TEM) micrograph of **1** on holey, carbon-coated copper grids (scale bar = 500 nm), shows nanorods in water at pH 8.5. Inset = high magnification of TEM image.

**Table 1.** UV/vis Absorption and Fluorescence Emission Data for OctaPhosPor **1** under Different pH Conditions in Water.

**pH**	**B-band (***λ***, nm; 10^5^ ɛ, M^−1^ cm^−1^)**	**Q-bands (λ, nm; 10^3^ ɛ, M^−1^ cm^−1^)**	**emission (*λ*, nm)**
3	442 (1.4)	516 (9.6), 656 (36)	no^[a]^
5	440 (2.19)	534 (21.2), 594 (14.8), 644 (12.8)	657, 721^[b]^
8	420 (2.38)	516 (13.8), 559 (12.8), 583 (12.0), 636 (10.6)	651, 718
10	418 (2.56)	510 (13.8), 545 (12.8), 578 (12.0), 626 (10.6)	651, 718

[a] very weak emission;

[b] weak emission.
